This article has been retracted.

# miR-15b represses BACE1 expression in sporadic Alzheimer’s disease

**DOI:** 10.18632/oncotarget.21177

**Published:** 2017-09-21

**Authors:** Guohua Gong, Fengmao An, Yu Wang, Ming Bian, Li-Jun Yu, Chengxi Wei

**Affiliations:** ^1^ Medicinal Chemistry and Pharmacology Institute, Inner Mongolia University for The Nationalities, Tongliao, Inner Mongolia, P.R. China; ^2^ Inner Mongolia Key Laboratory of Mongolian Medicine Pharmacology for Cardio-Cerebral Vascular System, Tongliao, Inner Mongolia, P.R. China; ^3^ First Clinical Medical of Inner Mongolia University for Nationalities, Tongliao, Inner Mongolia, P.R. China

**Keywords:** alzheimer’s disease, miR-15b, BACE1, cell viability, cell apoptosis

## Abstract

Beta-site Amyloid precursor protein Cleaving Enzyme 1 (BACE1) is conceived as a potential target for therapies against Alzheimer disease (AD). MicroRNAs (miRNAs) are small non-coding RNAs that negatively regulate gene expression in a sequence-specific manner. Although miRNAs have been increasingly recognized as important modulators in sporadic AD. In order to confirm whether miR-15b correlates with the BACE1 upregulation in sporadic AD, we firstly evaluated the expression of miR-15b and BACE1 in sporadic AD brain tissues and analyzed the correlation of miR-15b with BACE1. Then we determined the regulation of miR-15b in SH-SY5Y cells on the BACE1 expression. And finally we determined the targeting to 3’ UTR of BACE1 by miR-15b by a luciferase reporter. Downregulation of miR-15b alleviated Aβ-induced viability inhibition and decreased apoptosis in SH-SY5Y cells. Our results demonstrated that miR-15b play an important role in the cellular AD phenotype and might be involved in the pathogenesis of AD.

## INTRODUCTION

Alzheimer’s disease (AD) is a neurodegenerative disorder characterized by progressive memory loss and increasing dysfunction in mental behavior. AD presents an increasing clinical challenge in terms of diagnosis and treatment [1, 2]. Although progress has been made in identifying genes associated with AD, the pathogenesis of AD have not been elucidated until now. Diagnostic neuropathological features including extracellular amyloid plaques consisting of deposits of beta-amyloid (Aβ), intracellular neurofibrillary tangles consisting of hyperphosphorylated tau protein, and neuronal cell loss [3]. The β-site APP-cleaving enzyme 1 (BACE1) is validated as Alzheimer’s β-secretase and a therapeutic target for AD.

MiRNAs are endogenous non-coding 19-23 nucleotide long RNA molecules that are located on chromosome 1p22 [4]. It has been revealed that miRNAs can affect various physiological and pathological processes including AD [4, 5]. Recently, several miRNAs have been found to be related to AD pathogenesis by regulating the function of AD-relevant molecules [6, 7]. MicroRNA-15 (miR-15) family includes miR-15a, miR-15b, and miR-192, etc [8, 9]. MiR-15b has been implicated as a mediator of apoptosis by targeting the antiapoptotic gene *bcl*_*2*_ in mesenchymal stem cells and rat hepatic cells [10]. However, little is known concerning its potential role in AD development and progression. In this study, we sought to assess the function and molecular mechanisms of MiR-15b in AD. We found that MiR-15b expression is downpregulated in in a cellular AD model of primary neurons. We demonstrated that MiR-15b-mediated pathogenesis of AD was through the pathways of BACE1.

## RESULTS

### miR-15b expression is decreased in AD brains

We first examined miR-15b expression levels in 40 AD brain tissues by performing quantitative real-time PCR (qRT–PCR) analysis. The results revealed that miR-15b expression levels were significantly lower in sporadic AD brain tissues when compared with those in brain specimens from other subjects (Figure 1A; *P* < 0.01). Furthermore, to understand the significance of BACE1 expression in AD brain samples, we quantified the BACE1 mRNA level in sporadic AD brain tissues by qRT-PCR. As shown in Figure 1B, there was a significantly higher level of BACE mRNA in AD brains samples compared with the control group (*P* < 0.01). Then, we analyzed the BACE1 protein level in the sporadic AD brain samples by the western blot assay. We also found that BACE1 was significantly higher in AD group than in control group (Figure 1C). Then we determined the correlation of miR-15b and BACE1 level by Pearson’s correlation test. It was shown that the miR-15b level was negatively correlated with BACE1 expression in AD brain tissues (R = -0.343, *P* < 0.01).

**Figure 1:** The relative expression of miR-15b and BACE1 were determined by qRT-PCR and western blot in AD patients **(A)** miR-15b expression levels were significantly lower in sporadic AD brain tissues than control tissues. **(B)** BACE mRNA expression levels were significantly higher in sporadic AD brain tissues than control tissues. **(C)** BACE1 protein expression levels were significantly higher in AD group than in control group.

### miR-15b regulates Aβ-induced viability inhibition and apoptosis of SH-SY5Y cells

Aβ can suppress viability and induce apoptosis of neural cells, which may be involved in the initiation of AD pathology. The MTT assay was performed to assess the potential biological function of miR-15b in Aβ-induced viability inhibition of SH-SY5Y cell lines. MTT assay results showed that Aβ inhibited the viability of SH-SY5Y cells and downregulation of BACE1 enhanced the inhibitory effects of Aβ (Figure 2A). Downregulation of miR-15b relieved Aβ-induced viability inhibition of SH-SY5Y cells (Figure 2B). Moreover, flow cytometric analysis was utilized to investigate whether apoptosis regulation is a potential contributing factor to cell viability regulated by miR-15b. Flow cytometric analysis results showed that Aβ-induced apoptosis of SH-SY5Y cells and downregulation of BACE1 enhanced the induced effects of Aβ (Figure 2C). Downregulation of miR-15b decreased apoptosis of SH-SY5Y cells in the presence of Aβ (Figure 2D). This observation suggested that miR-15b might be an important regulatory factors in Aβ-induced viability inhibition and apoptosis of SH-SY5Y cells.

**Figure 2:** **(A)** MTT assay results showed that Aβ inhibited the viability of SH-SY5Y cells and downregulation of BACE1 enhanced the inhibitory effects of Aβ. **(B)** Downregulation of miR-15b relieved Aβ-induced viability inhibition of SH-SY5Y cells. **(C)** Flow cytometric analysis results showed that Aβ-induced apoptosis of SH-SY5Y cells and downregulation of BACE1 enhanced the induced effects of Aβ. **(D)** Downregulation of miR-15b decreased apoptosis of SH-SY5Y cells in the presence of Aβ.

### miR-15b regulates BACE1 expression by directly targeting BACE1 mRNA 3′-UTR

To address the roles of miR-15b in the AD pathology, we used web-based miRNA target prediction programmes TargetScan, PicTar, and miRanda to identify a gene of which 3′-UTR could match miR-15b. BACE1 is one of the candidates because miR-15b includes its potential binding sequences of the BACE1 mRNA 3′-UTR (Figure 3A). To test whether BACE1 is a functional target of miR-15b, we transfected a firefly luciferase reporter vector containing the wild-type (WT) binding site or mutant (MUT) site within the 3′-UTR of BACE1 into HEK293 cells. Overexpression of miR-15b, but not miR-control, decreased luciferase activity in cells transfected with luciferase reporter vector containing the WT 3′-UTR of BACE1. The luciferase activity was not affected in the cells transfected with luciferase reporter vector (control vector) or luciferase reporter vector containing the MUT 3′-UTR of BACE1 (Figure 3B).

**Figure 3:** MiR-15b regulates BACE1 expression by directly binding to the 3′-UTR of BACE1 mRNA **(A)** The putative binding sites of miR-15b in the wild-type 3′-UTR of BACE1 (BACE1 3′-UTR-WT) and mutated target sites of BACE1 (BACE1 3′-UTR-MUT). **(B)** Relative luciferase activity in HEK293 cells co-transfected with pGL3-BACE1–3′-UTRWT/MUT and miR-15b mimics or miRNA scramble control (miRcon).

To further validate whether miR-15b reduces the expression levels of BACE1, we determined the changes of BACE1 mRNA and protein using qRT-PCR and western blotting in SH-SY5Y cells transfected with miR-15b mimics or inhibitors. The qRT-PCR results showed that the levels of BACE1 mRNA were significantly reduced in cells transfected with miR-15b mimics, and inhibition of miR-15b could increase the levels of BACE1 mRNA (Figure 4A; either *P* < 0.05). The western blotting results indicated that the levels of BACE1 protein were negatively regulated by miR-15b (Figure 4B). These results suggest that miR-15b reversely regulates BACE1 expression by directly targeting the 3′-UTR of BACE1 mRNA.

**Figure 4:** The relative levels of BACE1 mRNA and protein in SH-SY5Y cells transfected with miR-15b mimics, miRNA mimic negative control (miR-con), miR-15b inhibitors (anti-miR-15b), or miRNA inhibitor negative control (antimiR-con) **(A)** The relative levels of BACE1 mRNA was measured using qRT-PCR after 48 h posttransfection.**(B)** The relative levels of BACE1 protein was measured using western blotting after 48 h posttransfection. Data are shown as means ± standard deviation (SD). **P < 0.01.

## DISCUSSION

Alzheimer’s disease (AD) is clinically characterized by deterioration of memory and cognitive functions, progressive impairment of daily living activities, and neuropsychiatric symptoms [12]. It was reported that the continuous production, degradation and the aggregation of Aβ lead to AD [13]. BACE1 is responsible for β-secretase activity, the rate-limiting step in the generation of Aβ. BACE1 is the rate limiting enzyme in the generation of Aβ from AβPP, and leads to the majority of Aβ production in AD pathology [14]. However, the underlying mechanisms of AD at the cell and molecular levels are still not completely elucidated.

More recently, a growing number of researches have focused on the regulatory roles of miRNAs [15]. MiRNAs have been reported to exert the biological function through regulating gene expression in AD patients [16, 17]. MiR-15b, a member of miR-15/16 family, has been implicated as a mediator of various diseases [18]. The gene encoding miR-15b itself is located in a cluster with miR-16-2. [19]. A recent study indicated that miR-16 is a good candidate for future drug development by targeting endogenous regulators of Aβ and Tau [9]. However, the molecular mechanisms by which miR-15b regulates AD biomarkers deserve further scrutiny.

In present study, we demonstrated significantly decreased expression of miR-15b and upregulation of BACE1 in AD brain tissues. There was a negative correlation of miR-15b and BACE1 in AD. We then investigated the negative regulation of miR-15b on the BACE1 expression in SH-SY5Y cells. The manipulated upregulation of miR-15b significantly downregulated the expression of BACE1 in both mRNA and protein levels in SH-SY5Y cells. Moreover, we demonstrated that BACE1 is a direct target of miR-15b, and BACE1 expression was regulated by miR-15b in HEK293 cells. Our findings may illuminate a mechanism by which miR-15b links to AD pathogenesis.

Abundant evidence demonstrates that direct toxicity of Aβ could contribute to the neuronal dysfunction and loss in AD. Apoptotic and cytoactive analyses of neurons indicated that Aβ decreased viability and induced apoptosis of neurons *in vitro*. In our study, Aβ inhibited the viability of SH-SY5Y cells and downregulation of BACE1 enhanced the inhibitory effects of Aβ. In addition, downregulation of miR-15b relieved Aβ-induced viability inhibition of SH-SY5Y cells. MiR-15b can supress the functions of SH-SY5Y cells, such as apoptosis and cell viability.

Our results demonstrated that miR-15b play an important role in the cellular AD phenotype and might be involved in the pathogenesis of AD. Based on these results, we propose the existence of a molecular event that may explain the pathogenesis of AD. However, further assays should be performed to verify the role of miR-15b *in vivo*.

## MATERIALS AND METHODS

### Human brain tissue

40 AD patients and 35 control subjects were implicated in this study. Frozen tissue samples of frontal cortices from autopsied and histopathologically confirmed AD and control cases were obtained from the University General Hospital. Each tissue sample was homogenized to 10% (w/v) final concentration in ice-cold 1x phosphate buffer solution (PBS), supplemented with Ribonu-clease inhibitor (Takara, Tokyo, Japan) and protease inhibitor cocktail (Roche Diagnostics, GmbH, Germany). And each homogenized sample was used for cellular extraction for mRNA, miRNA and protein. Prior to the operation, patients granted consent for the use of the excised brain tissue in medical or scientific research. And the use of frozen human brain tissue was approved by the Institutional Review Board of the Inner Mongolia University for the Nationalities.

### Cell culture and treatment

Human neuroblastoma SH-SY5Y cells and human embryonic kidney 293 cells (HEK293) were provided by the cell resource center of Chinese academy of medical sciences (Beijing, China). Cells were cultured in Dulbecco’s modified Eagle’s medium (DMEM) (Invitrogen, Carlsbad, CA, USA) containing 10 % heat-inactivated fetal bovine serum (FBS; Invitrogen), 100 units/ml penicillin, and 100 μg/mL of streptomycin (Sigma-Aldrich, St. Louis, USA) in a 37 °C and 5 % CO2 incubator. To obtain the neurotoxic form of Aβ, Aβ42 (Sigma-Aldrich) solution was keep at 37 °C for 4 days to induce an aggregated form of Aβ42 according to the methods described previously [11]. The aggregated form of Aβ42 was used at a final concentration of 10 μM. Twenty-four hours after transfection, SHSY5Y cells were subjected to Aβ treatment for 24 h. Cell viability and apoptosis were determined using 3-(4,5-dimethylthiazol-2-yl)-2,5-diphenyltetrazolium bromide (MTT) assay and flow cytometric analysis, respectively.

### Transfection

miR-15b mimics, miRNA mimic negative control (miRcon), miR-15b inhibitors (anti-miR-15b), and miRNA inhibitor negative control (anti-miR-con) were purchased from GenePharma (Shanghai, China). Synthetic miR-15b mimics, miR-con, miR-15b inhibitors, and anti-miR-con were transfected into cells using Lipofectamine 2000 (Invitrogen) according to the manufacturer’s instructions. Small interfering RNA (siRNA) vectors targeting BACE1 were purchased from GenePharma (Shanghai, China). Transfection was conducted using Lipofectamine 2000 (Invitrogen) according to manufacturer’s instructions.

### Quantitative real-time PCR

Total RNA and miRNAs were isolated using Trizol reagent (Invitrogen) and mirVana miRNA isolation kit (Ambion, Austin, TX, USA). Then cDNA was obtained by using oligo-dT primers or stem-loop reverse transcriptase (RT) primers, respectively. β-actin and U6 were used as controls for BACE1 and miR-15b, respectively. PCR was performed under the following conditions: 94°C for 4 min followed by 40 cycles at 94°C for 1 min, 56°C for 1 min and 72°C for 1 min. Relative expression levels of the genes were calculated using the 2^-ΔΔCt^ method.

### Western blot assay

At the indicated times (at 48 h after transfection), cells were harvested in ice-cold PBS and lysates were prepared by RIPA buffer (Beyotime, China). Protein concentration was determined by BCA Protein Assay Kit (Beyotime, China) at 570 nm. Equal amounts of protein were separated by 8% or 15% SDS–PAGE gels. Then gels were transferred onto polyvinylidene fluoride (PVDF) membranes (Millipore, Billerica, MS, USA). Furthermore, for immunoblot experiments, the membranes were blocked for 2 h with 5% nonfat milk in Tris-buffered saline containing 0.1% Tween-20 (TBST and were incubated with primary antibodies at 4°C over night. In addition, membranes were incubated with HRP-conjugated secondary anti-mouse or anti-rabbit antibodies (Multi Sciences, China) for 1 h at room temperature after washing. At last, membranes were visualized by a commercial enhanced chemiluminescent substrate (Bio-Rad, USA), and Image J was used to quantitate the expression of proteins.

### Luciferase reporting assay

The 3’ UTR of BACE1 and the CMV promoter were amplified from human chromosomal DNA and pcDNA3.1 (+) and cloned into the pGL3-luciferase basic vector (Promega, Madison, WI, USA). Sequences of primers and cloning strategy are available on request. For the luciferase assays, 50 nM of miR-16b mimics or scrambled RNA were co-transfected with the reporter vector and the Renilla control vector (Promega, Madison, WI, USA) into the HEK293 cells by Lipofectamine 2000 (Invitrogen, Carlsbad, CA, USA). 24 h post transfection, the measurements were performed using the Dual luciferase re-porter assay kit (Promega, Madison, WI, USA). Or the HEK293 cells post the transfection for 24 h was lyzed for western blot analysis.

### Statistical evaluation

Each experiment was performed as least three times and the data are expressed as the mean ± standard error. For the analysis of miR-15b and U6, BACE1 and β-actin in mRNA or in protein level in protein level, between two groups, and data were analyzed using the Student’s t test. The nonparametric Pearson’s correlation test was performed to evaluate the correlation of miR-15b with the BACE1 mRNA level. A statistical significance was considered when *P* < 0.05. *P*<0.05 was considered to indicate a statistically significant difference. All statistical analyses were performed using the SPSS 10.0 statistical software package (SPSS, Inc., Chicago, IL, USA).
